RETRACTED

# Application of Calcium-Based Nanomaterials in Art Sculpture Reinforcement Technology

**DOI:** 10.1155/2022/9593268

**Published:** 2022-10-04

**Authors:** Kun Di

**Affiliations:** Xi'an Academy of Fine Art, Xi'an, Shaanxi 710000, China

## Abstract

In order to solve the problem of the reinforcement effect of art sculpture, the author proposes the application of a calcium-based nanomaterial in the reinforcement process of art sculpture. This application mainly passes the unconfined compression test, direct shear test, penetration resistance test, and disintegration test, and an in-depth evaluation of the reinforcement effect of different calcium-based reinforcement agents on the site soil was carried out from the perspective of mechanical strength and water stability. The results showed the following: Compared with the untreated samples, the unconfined compressive strength of the samples treated with nano-calcium oxide and nano-calcium hydroxide increased by 13.5% and 25.9%, respectively, and the cohesion increased by 69.8% and 97.7%. *Conclusion*. Calcium-based nanomaterials fill in the pores between soil particles to support the soil particles, which greatly improves the mechanical strength and water stability of the specimen.

## 1. Introduction

With the continuous improvement of social and economic levels, people are more and more thirsty for spiritual culture; they also put forward higher requirements for urban cultural construction, and public art sculpture is a part of urban cultural construction. Ceramic sculpture is an indispensable part of urban public art [1]. Artists make clever use of ceramic materials, and the aesthetic concepts in modern society and the thoughts and emotions between man, nature, and society are fully expressed through a unique language and culture of the soil, forming a unique modern ceramic art culture [2]. With the continuous development of modern ceramics, public art works with ceramics as the main material have emerged, and with the corrosion resistance and other characteristics of ceramic materials, they gradually present a scene of prosperity and development, and works of art are no longer decorations that exist in the interior. They appear in the public environment with a brand-new image and are skillfully integrated with the surrounding buildings, people, local historical changes, humanistic culture, etc., forming an artistic beauty with a unique flavor [3].

Modern ceramic sculpture has an extraordinary position in urban public art in different types and expressions, and through the mutual connection of information transmission and the mutual cooperation of emotional expression between works, the overall image of a city can be effectively improved, thereby increasing the city's popularity and attracting people from all over the world to come and watch. This will help to promote the development of tourism in the city, improve the economic level of the city, and realize the effective integration of the city's historical culture, humanistic heritage, modern urban architecture, and development, to enhance the external image of the city and beautify the internal cultural environment of the city [4].

RETRACTED

A public art sculpture is a sculpture with an artistic nature in public space [5]. Public art can exist in different forms due to different environments, and the meaning of public art sculptures is also different, which will be consistent with the urban public environment [6]. Incorporating the spirit of the public environment into the design of public art sculptures and transforming public art into regional cultural symbols can have a certain impact on the urban environment and audience [7]. Ceramic sculpture is an indispensable part, the use of ceramic materials in public art sculpture can make more people pay attention to traditional Chinese culture, more cultural connotations and humanistic thoughts are conveyed through ceramic sculptures, and through the different characteristics of ceramic materials, targeted design of different forms of ceramic art can be created [8]. In the broad and profound cultural river, the development of ceramic sculpture has also shown a prosperous trend with the wide application of modern ceramic art [9]. For the research of ceramic sculpture, we still need to constantly ponder and explore, as shown in Figure 1:

## 2. Literature Review

In the past ten years, thanks to the rapid development of materials engineering and biological science, the use of calcium carbonate deposits to improve the mechanical properties and stability of rock and soil is a hot topic in current research [10]. At present, there are three main methods of calcium carbonate deposition: chemical synthesis, biomineralization, and biomimetic mineralization; the corresponding typical methods are in situ calcium carbonate deposition (CIPS), microbial-induced calcium carbonate, deposition method (MICP), enzyme-induced calcium carbonate deposition method (EICP), etc.

Limewater is a traditional inorganic reinforcement material, which was used in the weatherproof reinforcement projects of stone cultural relics in England as early as the early 19th century [8]. As an air-hardening building material, lime can react with CO_2_ in the air to form CaCO_3_ deposition [11]. Although this method was tried very early, it was eventually discontinued due to the unsatisfactory reinforcement effect [12]. However, cultural relics protection scientists did not give up research on lime curing agents [13]. With the rapid development of nanotechnology, appropriate modification of traditional materials, with the help of special quantum effects, surface effects, and local field effects of nanoparticles, enables them to exhibit a series of properties different from ordinary crystalline and amorphous substances, making them better meet the requirements of cultural relics protection [14]. The development and application of nano-calcium hydroxide reinforcement abroad have been relatively advanced [15]. There are many laboratories that can prepare nano-calcium hydroxide in small batches and optimize it according to the characteristics of the reinforcement object, and some companies have launched a series of nano-calcium hydroxide curing agents with excellent performance [16].

RETRACTED

Based on the above-mentioned several mainstream calcium deposition methods, the potential and feasibility of weatherproof reinforcement on the surface of soil sites are discussed from the aspects of the reinforcement itself, reinforcement mechanism, and potential risks [17]. CIPS reinforcement has a very low viscosity coefficient, and at the same time, the consolidation time is adjustable, and it has good reinforcement depth and curing strength, but it is sensitive to ambient temperature; in actual use, the composition of the reinforcement liquid needs to be adjusted according to the preset temperature optimization [18]. Due to their many by-products, most of them are soluble inorganic salts, although most of these inorganic salts will be gradually lost with the water cycle when they are used for the reinforcement of ordinary sandy soil; too many soluble salts for soil sites will eventually be enriched in the surface layer of the site, which may accelerate the weathering of the site [19]. Relying on the nanoscale particle size and extremely high reactivity, the nano-calcium hydroxide reinforcement greatly improves the penetration ability and reinforcement performance of traditional lime water and improves the application effect of calcium hydroxide reinforcement materials in the protection of cultural relics.

## 3. Methods

### 3.1. Test of Basic Properties of Soil for the Test

The soil used in this test was taken from the ancient wave section of the Ming Great Wall in a certain place, the complete block soil samples that fell off the body were selected, the surface weathering layer was removed, and the soil samples were properly sealed on-site to avoid soil damage and basic parameter changes during transportation.

The basic parameters of the soil tested included the following: moisture content, density, specific gravity of soil particles, particle curve, limit moisture content, compaction test, and chemical composition analysis of soluble salts. The test methods used in each test are shown in Table 1.

RETRACTED

#### 3.1.1. Determination of Moisture Content

Moisture content is one of the basic physical property indexes of soil. It directly reflects the state of the soil, and the change in the moisture content has a significant impact on the physical and mechanical properties of the soil. During the test, the soil samples were placed in an oven, and the temperature was set at 105°C until the weight was constant and then weighed. Generally, the soil samples used in this experiment have little difference in moisture content, ranging from 1.5 to 2.1%.

#### 3.1.2. Density Measurement

The density of soil reflects the compactness of the soil and is a necessary parameter to convert the dry density, porosity, and void ratio of soil. From the test results, the samples used in the test have large differences in density due to the difference in weathering degree and sampling location, and the variation range of dry density is 1.52 − 1.66 g/cm^3^.

#### 3.1.3. Determination of Specific Gravity of Soil Particles

The specific gravity of soil is the average value of the specific gravity of various minerals in the soil, which is related to the types and contents of minerals that make up the soil and is also an important basis for calculating porosity, void ratio, and saturation. The calculation formula is as follows:

(1) $$\begin{array}{c} G_{s}=\frac{m_{d}}{m_{1}+m_{d}-m_{2}}\cdot G_{wT}. \end{array}$$

In the formula, *G*_s_ is the specific gravity of the soil particles; *m*_d_ is the mass of the dried soil particles; *m*_1_ is the mass of the pycnometer plus water; *m*_2_ is the total mass of the pycnometer, water, and the sample; and *G*_*wT*_ is *T*°*C*, the specific gravity of pure water or neutral liquid.

After calculation, the average specific gravity of soil particles in this batch of test soil was 2.71.

#### 3.1.4. Particle Analysis and Determination

From the results of the particle test (Table 2), the particle size is mainly concentrated in the 0.075 ~ 0.005mm range; this included mainly powder particles, containing a certain amount of clay (18.92%), with the nonuniformity coefficient *C*_*ll*_=8.99 and the curvature coefficient *C*_*c*_=1.28, and it can be concluded that the soil of this site is well-graded soil.

#### 3.1.5. Determination of the Limit Moisture Content

With the change in moisture content, soil can have four states, namely, solid state, semisolid state, plastic state, and flow state. The critical moisture content of soil transition from one state to another state is defined as the limit moisture content. According to the different transformation states, the limit water content can be divided into liquid limit *ω*_*L*_, plastic limit *ω*_*P*_, shrinkage limit *ω*_*S*_, and so on. In addition, the difference between the liquid limit and the plastic limit is defined as the plasticity index *I*_*P*_.

RETRACTED

The combined liquid-plastic limit determination method was adopted for the soil used in this experiment (Figure 2). It was concluded that the plastic limit of the Gulang section of the Ming Great Wall site was 17.4%, the liquid limit of 17 mm was 30.4%, and the plasticity index was 13. According to the relationship between the plasticity degree and liquid-limited clay content (Table 3), it can be found that the site soil is medium plastic soil.

#### 3.1.6. Determination of the Optimal Moisture Content

The main purpose of the compaction test is to measure the maximum dry density and optimum moisture content of the disturbed soil, understand the compaction characteristics of the soil, and provide a basis for the configuration of moisture content in the subsequent sample preparation. Its optimum moisture content is about 16.8%, and its maximum dry density is 1.69 g/cm^3^, showing typical silt characteristics.

#### 3.1.7. Determination of Soluble Salt Content

The overall soluble salt content of the soil samples from the site is relatively high; from the perspective of single ion species, the content of sulfate ions, calcium ions, sodium ions, and potassium ions is relatively high.

### 3.2. Specimen Preparation

This experiment covered both the remodeled and undisturbed samples. By selecting the reshaped sample, the basic parameters such as dry density and moisture content of the sample can be controlled artificially, so that the reinforced sample and the unreinforced sample have the same initial state and mechanical properties and the comparability of the test results is enhanced. In the process of the water stability test, since the cementation state and stress history between the particles of the remodeled soil are essentially different from those of the actual site soil, in order to more objectively reflect the change of water resistance after reinforcement treatment in the actual state, the undisturbed samples cut into blocks of the same sample were selected for disintegration testing.

The preparation of indoor remodeling samples was based on the measured density of soil samples under moderate weathering degrees, and the dry density was controlled at 1.5 g/cm^3^. The remodeling sample preparation utilizes the principle of static compaction and adopts the site soil remodeling sample-making machine designed by a research institute; the sample making machine adopts a double-sided compaction design, which solves the defect of uneven compactness of the compression surface and bottom surface of the sample caused by single-sided compression in the past. The specific preparation process is as follows: The undisturbed rammed earth was crushed and passed through a 2 mm sieve, and distilled water was added to form a wet soil with a moisture content of 14%; after sealing with a plastic bag, it was placed in a humidifier for 24 hours to allow the water to be dispersed evenly. Specimens of 5 cm × 5 cm × 5 cm size were used for the determination of unconfined compressive strength, and specimens of 7.07 cm × 7.07 cm × 7.07 cm size were used to prepare ring knife specimens for the direct shear test; the inner diameter of the ring knife is 6.18 cm, and the height is 2.0 cm. The sample of the ring knife is cut from the middle of the square sample. After the sample preparation is completed, it is placed in a laboratory environment to dry naturally.

RETRACTED

The undisturbed soil sample used for the disintegration test is selected with a more regular shape, and the rammed earth with a uniform weathering degree and no crack development is cut into four undisturbed cubes with side lengths of 3.0 ± 0.3 cm, as a set of samples; the purpose is to make the properties of the four samples as similar as possible. In the same way, the remaining undisturbed rammed earth is cut in this way, and the prepared undisturbed cubes are classified into groups of four for subsequent water stability testing.

### 3.3. Reinforcement Method

In order to ensure sufficient calcium absorption and avoid the phenomenon of white hair on the surface, the reinforcement method of low concentration and multiple penetrations is adopted. The nano-calcium oxide calcined at 800°C and the nano-calcium hydroxide prepared by the microemulsion method were selected as the nano-calcium-based materials, calcium oxide (AR) was used as the calcium-based comparative material, and the design concentration was 10 g/L; at the same time, we set the reference group without any reinforcement. The infiltration amount of the single reinforcement is determined by the maximum saturation *Sr*=65%, and the single reinforcement amount is given in

(2) $$\begin{array}{c} S=\left(1-\frac{\rho_{d}}{G_{s}\rho_{w}}\right)\cdot V\cdot Sr. \end{array}$$

In the formula, *S* is the volume of single reinforcement liquid, cm^3^; *ρ*_*d*_ is the dry density of the soil sample, 1.5 g/cm^3^; *G*_*s*_ is the specific gravity of soil particles, which is 2.71; *ρ*_*w*_ is the density of water, which is 1.0 g/cm^3^; V is the total volume of the sample, cm^3^; and *Sr* is 0.65.

RETRACTED

The reinforcement process of various types of samples is shown in the Table 4. After the samples are reinforced, they are placed in a curing box with constant temperature and humidity, and relevant mechanical and water stability tests are carried out after curing for 28 days.

### 3.4. Test Method

#### 3.4.1. Unconfined Compressive Strength Test

Unconfined compressive strength *q*_*u*_ is a common index among soil strength indexes and is easy to measure. The test uses an electrohydraulic servo universal testing machine with a controlled loading speed of 1.0 mm/min; 4 samples are set in each group, and the average value is taken as the compressive strength. After each sample was damaged, an appropriate number of soil samples were taken for moisture content determination.

#### 3.4.2. Direct Shear Test

The author used a ZJ-type strain-controlled direct shearing instrument to set 4 samples in each group and consolidated them under vertical pressures of 100 kPa, 200 kPa, 300 kPa, and 400 kPa, respectively, until the deformation was stable; a horizontal shear force was then applied at a shear rate of 0.8 mm/min until the sample was sheared.

#### 3.4.3. Drilling Resistance Test

The micro-damage drilling resistance system was independently designed by the cultural relics protection research center of a certain university. The parameters of this test were set as follows: the diameter of the drill bit was 2 mm, the rotation speed was 1000 rpm, the drilling rate was 0.2 mm/s, and the drilling depth was 20 mm. The sample was fixed, the center of the infiltration surface was facing the drill bit, and the position of the drill bit was adjusted so that the drill bit was in slight contact with the top surface of the sample.

#### 3.4.4. Disintegration Test

The water stability of soil is closely related to the internal structure of soil and the form of cementation between soil particles. Improving the water resistance of soil after reinforcement is an important index to evaluate the effectiveness of reinforcement materials. According to the requirements of the disintegration test specification, the original samples were selected to test the samples before and after reinforcement. It can be considered that the properties of the four samples in the same group are similar, treated with calcium oxide (AR), nano-calcium oxide, and nano-calcium hydroxide reinforcements, respectively, while leaving the sample without any treatment. The test steps are as follows: first place a group of four samples on a metal mesh frame, add a sufficient amount of distilled water to the container, then put the metal mesh frame into the container horizontally, and keep the top surface of the sample submerged about 1 cm below the liquid surface, so that there is enough space between the bottom of the sample and the bottom surface of the container. During the whole process, a digital camera was used to shoot the whole process; after the test, the disintegration process and form of the sample were recorded according to the video playback, and the video pictures were intercepted for related comparison.

RETRACTED

## 4. Results and Discussion

According to the requirements of the reinforcement materials for the protection of cultural relics, the selected reinforcement agent should try not to change the original color of the cultural relics. During this test, the color change of the sample surface was observed. During the dropping process of the nano-calcium-based material, there is no significant difference between the samples treated with different reinforcement agents. In the later drying process, the samples after reinforcement treatment can be clearly observed, and with the volatilization of the solvent, the “whitening” becomes more and more obvious. Taking the sample used for the direct shear test after curing as an example, it is found by comparison that, after ordinary calcium oxide (AR) reinforcement, the surface of the sample is significantly white, the surface layer is in a state of fine shelling, and the powder falls off by gently sliding it with the fingers. The surface of the sample treated with nano-calcium oxide and nano-calcium hydroxide reinforcement also has a certain “whitening” phenomenon, but the surface of the sample is smoother than that of the unreinforced sample, and there is no pulverization phenomenon. The surface is swiped with the fingers, and it is noted that no soil particles fall off. However, in general, the surface whitening phenomenon is still relatively serious, and related improvement in materials or reinforcement methods is still required in the later stage.

Compared with the unreinforced samples, the moisture content of the samples in the natural air-dried state after infiltration and reinforcement of calcium-based materials is slightly lower. From the point of view of compressive strength, the samples after infiltration treatment with calcium oxide (AR) reinforcement liquid showed a certain loss of strength. The strength of the samples treated with the nano-calcium oxide reinforcement solution and the nano-calcium hydroxide reinforcement solution increased by 13.5% and 25.9%, respectively. It can be considered that the untreated calcium oxide (AR) reinforcement liquid is relatively large due to its large dispersed particles; it cannot easily enter the interior of the sample, and at the same time, the sample swells slightly under the immersion of the reinforcement solution, and the spacing between soil particles increases, which is the reason why the strength does not increase but decreases after reinforcement. Although the swelling effect still exists after the treatment of the nano-calcium oxide reinforcement solution and the nano-calcium hydroxide reinforcement solution, as the nano-calcium-based material enters the soil sample, filling between soil particles forms an effective cementation mechanism, which improves the strength. Due to its larger specific surface area and reactivity, the reinforcement effect of nano-calcium hydroxide has been further improved on the basis of nano-calcium oxide.

RETRACTED

Figures 3(a) and 3(b) show the shear stress-shear displacement curves of the reinforced and unreinforced specimens. From the relationship between shear stress and shear displacement under different vertical pressures, the following laws exist: under a vertical pressure of 100 kPa (Figure 3(a)), after the unreinforced sample experienced a brief elastic deformation stage in the initial stage and after the shear displacement reaches 2.0 mm, the growth of shear stress tends to ease, but it maintains a slight increase does not converge until the end of the test, showing the characteristics of certain strain strengthening. The reinforced samples showed elastic deformation characteristics in the small shear displacement stage. The samples reinforced with calcium oxide (AR) first reached the peak shear strength of 1.2 mm, and then, the shear strength decreased to 1.8. The residual shear stage is entered when the shear displacement occurs; the samples treated with nano-calcium oxide and nano-calcium hydroxide reinforcement maintain approximate elastic deformation before the shear displacement of 0.6 mm and 1.3 mm, respectively, and reach peak strength at the shear displacement of 0.6 mm and 1.3 mm; the shear strength then decreased significantly and entered the shear yield stage at a shear displacement of 2 mm. Under the vertical pressure of 200 kPa, the law of shear stress and shear displacement reflected by the reinforced and unreinforced samples (Figure 3(b)) is basically similar to that under the vertical pressure of 100 kPa.

In addition, by comparing the shear stress-shear displacement relationship curves of the reinforced and unreinforced specimens, it can also be found that there are two obvious laws under vertical pressure at all levels: that is, the peak shear strength of the sample reinforced with nano-calcium hydroxide is the largest, followed by the sample reinforced with nano-calcium oxide and the sample after calcium oxide (AR) treatment, except for the slope of the small shear deformation stage. In addition to the difference from the unreinforced sample, there is no significant difference in its peak shear strength. From the point of view of the residual shear strength of the samples, the reinforced sample falls back after reaching the peak shear strength and the final residual shear strength is similar to that of the unreinforced sample. The peak shear strength and residual strength values of each group of samples are shown in Table 4.

RETRACTED

Figure 4 shows the variation law between the drilling resistance and the drilling depth of the samples treated with different calcium-based reinforcement agents, and the unreinforced samples were set as reference samples at the same time. It can be seen from the figure that the resistance value of the reshaped sample without reinforcement treatment is always small before the drilling depth of 7 mm, indicating that the surface layer is relatively loose and the cohesion between soil particles is low. The samples treated with nano-calcium oxide and calcium oxide (AR) reinforcement agent, compared with the untreated sample, entered the stage of rapid resistance growth (at 6 mm) earlier; from the growth trend of the curve, the curing effect of nano-calcium oxide and calcium oxide (AR) reinforcement is similar, and compared with the untreated sample, the improvement is not too obvious. The sample reinforced with nano-calcium hydroxide entered a rapid growth stage when it was drilled into about 2 mm, which indirectly reflected that the strength of the sample was significantly improved after being treated with nano-calcium hydroxide, the cohesion between soil particles was strengthened, and the average drilling resistance value was much higher than those of the other three groups of samples.

Compared with the untreated samples, the unconfined compressive strength of the samples treated with nano-calcium oxide and nano-calcium hydroxide increased by 13.5% and 25.9%, respectively, and the cohesion increased by 69.8% and 97.7%.

## 5. Conclusion

The author proposes the application of calcium-based nanomaterials in the reinforcement process of art sculpture and mainly discusses the test and evaluation of the reinforcement effect of nano-calcium-based materials on the soil of the site, mainly including color change observation, compressive strength test, direct shear test, penetration resistance test, and disintegration test, etc. From the indoor reinforcement test, the samples treated with nano-calcium hydroxide and nano-calcium oxide reinforcement, the mechanical properties and water stability are improved to varying degrees and the reinforcement effect of nano-calcium hydroxide is better than that of nano-calcium oxide reinforcement. Compared with the unreinforced samples, the samples after infiltration and reinforcement of nano-calcium-based materials have significantly improved in terms of mechanical strength and water stability and have a certain application potential for the reinforcement of soil sites in the arid environment of Northwest China.

RETRACTED

## Figures and Tables

**Figure 1:** Application of calcium-based nanomaterials in the reinforcement of art sculptures.

**Figure 2:** Limit moisture content of soil for the test.

**Figure 3:** Stress-strain relationship curves under different vertical pressures.

**Figure 4:** Drilling resistance curves of treated and untreated samples with different calcium-based reinforcements.

**Table 1:** Test methods used in various tests.

Serial number	Pilot projects	Experiment method
1	Moisture content test	Drying method
2	Density test	Wax seal
3	Soil grain specific gravity test	Pycnometer method
4	Particle analysis test	Decorative analysis
5	Limit moisture content test	Combined determination of liquid plastic limit
6	Optimum moisture content test	Light compaction
7	Soluble salt content test	Submit for inspection

**Table 2:** Particle size analysis.

1 ~ 0.5 mm	0.5 ~ 0.25 mm	0.25 ~ 0.1 mm	0.1 ~ 0.075 mm	0.075 ~ 0.005 mm	<0.005 mm	Unevenness factor *C*_*u*_	Curvature coefficient *C*_*c*_
0.22%	1.33%	3.87%	5.24%	70.42%	18.92%	8.99	1.28

**Table 3:** Relationship between plasticity degree of general soil and liquid limit clay content.

Plasticity of soil	No plasticity	Low plasticity	Mesoplastic	High plasticity
By plasticity index *I*_*P*_	<3	3 ~ 10	10 ~ 17	>17
By liquid limit *ωL*(%)	<20	20 ~ 30	30 ~ 40	>40
By clay content (%)	<6	6 ~ 15	15 ~ 30	>30

**Table 4:** Peak shear strength and residual strength values of each group of samples.

Types of reinforcement fluids	Maximum shear strength (kPa)				Residual shear strength (kPa)			
	100 kPa	200 kPa	300 kPa	400 kPa	100 kPa	200 kPa	300 kPa	400 kPa
Not processed	87.84	134.59	199.60	231.75	74.87	129.51	189.90	233.35
Calcium oxide (AR)	83.75	155.51	183.90	243.70	69.39	140.95	188.87	243.78
Nano-calcium oxide	104.08	184.43	226.42	259.29	71.21	131.47	199.03	241.30
Nano-calcium hydroxide	129.65	171.64	251.99	275.73	70.04	133.30	197.21	234.38

## Data Availability

The data used to support the findings of this study are available from the author upon request.
